RETRACTED

# Sports Training Strategy and Interactive Control Method Based on Digital Twins and Wireless Sensor Networks

**DOI:** 10.1155/2022/2131125

**Published:** 2022-06-16

**Authors:** Zheyu He, Xi He

**Affiliations:** ^1^Department of Physical Education, Sangmyung University, Graduate School, Seoul 03016, Republic of Korea; ^2^College of Physical Education, Qilu Normal University, Jinan 250013, Shandong, China

## Abstract

By combining virtual reality, the digital twin system has been deeply applied in many places. Especially with the upsurge of national sports and more attention to sports, people have also begun a more in-depth study on the strategy of sports training. This paper aims to explore the application of the Brazilian jujitsu training strategy and interactive control method in the new era. Based on the sports skills of Brazilian jujitsu, combined with digital twin technology and wireless sensor network technology, this paper develops a sports training system based on Brazilian jujitsu. It can collect the action information of the trainer and twin it into the simulation system so as to carry out better and more effective confrontation training. The experimental results show that the average delay time is 5.2 ms and the maximum delay time is 6.5 ms, which is less than the limit delay time of 20 ms. Compared with the control group, it achieved quite good results. It shows the effectiveness of the system designed in this paper for trick jujitsu training.

## 1. Introduction

With the rise of the digital twin concept, based on digital twin technology, this paper serves physical training. This paper aims to optimize the new mode of sports training strategy management and control, Digital twin training platform, which has gradually become the current development hotspot. Brazilian jujitsu “ground surrender” technology has increasingly highlighted its technical advantages and practical value in comprehensive fighting, jujitsu competitions, and other events. It is a technique of combining technology and theory, winning with skill and overcoming hardness with softness. It has many advantages in subduing opponents in the competition. In addition to standing confrontation, Brazilian jujitsu focuses more on ground fighting. Repeated actual combat confrontation is the basic training method of Brazilian jujitsu, which is a real fighting method. From the cultural perspective, Brazilian jujitsu, as a martial art that originated in the East and evolved under western culture, has a unique cultural connotation. Therefore, it is necessary to study this.

The conceptual framework of the digital twin and five-dimensional digital twin model have been proposed. However, based on it, this paper proposes a more comprehensive and detailed reconfigurable digital twin manufacturing system architecture for the operation and maintenance requirements and reconfiguration requirements of the digital twin manufacturing system. This paper aims to guide the construction of a digital twin manufacturing system with high fidelity, high practicability, high flexibility, intelligence, and reconfigurability. It enables it to give full play to the comprehensive advantages of big data based manufacturing, virtual manufacturing, and flexible manufacturing in the market competitive environment with rapid changes in products, technology, and demand.

RETRACTED

## 2. Related Work

Many scholars have their own views on the research of twins and wireless sensor networks. Lee proposed a unified three-tier blockchain architecture as a guideline for researchers and the industry. He clearly identified the potential of blockchain and adapted, developed, and integrated the technology with their manufacturing development to move towards industry 4.0 [1]. In order to realize the digital twin vision of health examination data, Li et al. constructed a general diagnosis and prognosis probability model by using the concept of a dynamic Bayesian network. He explained the proposed method through an example of fatigue crack propagation of aircraft wings [2]. Hammoudeh et al. considered wireless sensor networks (WSN) as a low-cost technology. It can provide intelligent LED solutions to effectively and continuously monitor large, busy, and complex landscapes. He proposed a method to calculate the number of sensor nodes to be deployed in order to achieve the specified coverage level according to the selected indicators in a given band area. It also maintains a radio connection within the network [3]. Zhao et al. combined the two sensors to receiver binding algorithms as an inner layer optimization to evaluate the fitness value of the solution. His experimental results showed that it is better than the existing methods. In addition, his method has good scalability, which can be used to deploy large-scale sensor networks [4]. Lamonaca F had proposed a program to overcome the inconvenience of data transmission. The new fully distributed and consensus based program iteratively filters the messages communicating with the NSN, which will increase the time delay within the allowable range. Therefore, the synchronization accuracy can be maintained regardless of the spatial distribution of ASN and NSN. He conducted numerical and experimental tests to verify the proposed procedure [5]. Edler et al. believed that project managers have the opportunity and professional responsibility to explore different curriculum models. He eventually developed better ways to train future sports coaches. In addition, educators have a responsibility to measure and report results to help provide a body of knowledge about best practices in clinical education [6]. However, the development and popularization of Brazilian jujitsu in China are not yet mature. Chinese experts and scholars have less research on the “ground surrender” technology of Brazilian jujitsu, and the basic theoretical research lacks breadth and depth.

RETRACTED

## 3. Digital Twins and Wireless Sensor Networks

### 3.1. Digital Twins

Brazilian jujitsu is also called Gracie jujitsu. It is a kind of martial arts that is good at sleeping skills, specializing in surrender, comprehensive fighting competition, and systematic defense [7, 8]. Jujitsu originated from the fighting on the ancient battlefield in Japan. After it was introduced into Brazil, it was developed into a new technical school by the Gracie family. Brazilian jujitsu is good at small, broad, and strong. Jujitsu practitioners often drag their opponents to the ground in combat. It uses lever force to form joint skills or twisting skills to subdue the opponent. The practice methods of Brazilian jujitsu can be divided into technical practice, independent practice, and confrontation practice. They often use technical exercises to improve their skill level and use independent exercises to improve their awareness of actual combat. It uses confrontation practice to enhance spiritual will.

Digital twin was first proposed by American professors in 2002 and was applied to product life cycle management at that time. After that, the concept of digital twins was noticed by the US Department of defense. NASA applied digital twins to the production and maintenance of spacecraft and flight training. Based on the physical entity of spacecraft, this paper constructs its virtual model. And it drives the operation of the virtual model through historical data and real-time collected data. Finally, it achieves the real mapping of the whole life cycle of the spacecraft in the virtual scene so as to realize the simulation prediction in the virtual environment.

In this paper, the digital twin system is used to simulate and reconstruct Brazilian jujitsu, which has multiple training advantages. As shown in Figure 1, the data twin reconfigurable system framework has a four-tier architecture, including the physical layer, model layer, service layer, and data layer.

### 3.2. Human Joint Twinning Algorithm

In order to meet the requirements of system flexibility, scalability, and telepresence [9], this paper uses Unity3D to design the virtual space part of the digital twin system. Unity3D is one of the most popular commercial game engines at present. It is famous for its realistic environment, good scalability, cross platform, and active software ecology. Its internal script is written in c# language [10]. This paper takes Brazilian jujitsu trainers as the research object and irb14000 dual arm cooperative robot as the simulation. The schematic diagram of the degree of freedom of the trainer's joint is shown in Figure 2.

RETRACTED

The joint angle corresponding to Figure 2 is shown in Table 1, and the motion range of each joint is shown in Table 2.

Virtual scene includes user interaction interface, virtual robot model, console and other virtual objects [11–13]. The standard model format in Unity3D is FBX, and the 3D model format of irb14000 officially provided by abb is STL format. Therefore, it is necessary to preprocess the model before importing the 3D model [14, 15]. The original model has too many triangular patches. This problem makes it difficult to load the model in Unity3D, which cannot achieve fluency and is not conducive to rendering. Therefore, this paper uses pixyz software to cut triangular patches of the original model. This paper specifies that each joint of the robot joint rotates around the *Z* axis of its parent object. In this paper, 3Dmax software is used to adjust the relationship between the joints and the rotation axis of each joint. It makes the parent of each joint of the joint its previous joint. The reason for this is that the child object needs to rotate with the parent object. Finally, the processed robot 3D model is exported to FBX format, and the adjusted joint hierarchical relationship is shown in Figure 3. The joints are connected by flanges, and the simulation control is arranged in the important order of 1 to 7 to complete the simulation control.

In vector calculus, the Jacobian matrix is a matrix whose first-order partial derivatives are arranged in a certain way, and its determinant is called the Jacobian determinant. The importance of the Jacobian matrix is that it embodies the optimal linear approximation of a differentiable equation and given points. The Jacobian matrix in robot space represents the relationship between joint velocity and end velocity. The expression of the end pose vector is as follows:

(1) $$\begin{array}{c} r={\left[x,y,z,\alpha ,\beta ,\gamma \right]}^{T}. \end{array}$$

*x*, *y,* and *z* are the ends of the joints. *α*, *β*, and *γ* identify the end posture of the joint, then the forward kinematics relationship of the joint can be obtained, as shown in the formula:

(2) $$\begin{array}{c} r=r\left(q\right). \end{array}$$

Among them,

(3) $$\begin{array}{c} q=\left[\theta_{1},\theta_{2},\theta_{3},\theta_{4},\theta_{5},\theta_{6},\theta_{7}\right]. \end{array}$$

Formula (3) represents the rotation vector of the joint, which can be obtained by time derivation:

(4) $$\begin{array}{c} v_{c}^{k}==\dot{r}=J\left(q\right)\dot{q}. \end{array}$$

Among them, *v*_*c*_^*k*^ is the spatial velocity including the translation velocity and rotation velocity components in the coordinate system *k*. *C* is the number of joints, and matrix *J* (*q*) is the mapping relationship between joint velocity and end velocity.

RETRACTED

According to formula (4), the relationship expression between joint speed and end speed of redundant joint can be obtained, as shown in the following formula:

(5) $$\begin{array}{c} \dot{q}=J{\left(q\right)}^{+}v. \end{array}$$

*J*(*q*)^+^ is the generalized inverse matrix of robot Jacobian matrix J(q), that is, the pseudoinverse used in this paper.

For the vector in three-dimensional space, it can be extended from the vector rotation of a two-dimensional plane, for the matrix *M*_*RX*_, *M*_*RY*_, *M*_*RZ*_ of *θ* the angle of rotation of the three-dimensional vector *ρ* around the *X* axis, *Y* axis, and *Z* axis in space, as shown in the following formulas:

(6) $$\begin{array}{c} M_{RX}=\left[\begin{array}{ccc} 1 & 0 & 0\\ 0 & \text{cos}\theta & -\text{sin}\theta \\ 0 & \text{sin}\theta & \text{cos}\theta \end{array}\right]. \end{array}$$

(7) $$\begin{array}{c} M_{RY}=\left[\begin{array}{ccc} \text{cos}\theta & 0 & \text{sin}\theta \\ 0 & 1 & 0\\ -\text{sin}\theta & 0 & \text{cos}\theta \end{array}\right]. \end{array}$$

(8) $$\begin{array}{c} M_{RZ}=\left[\begin{array}{ccc} \text{cos}\theta & -\text{sin}\theta & 0\\ \text{sin}\theta & \text{cos}\theta & 0\\ 0 & 0 & 1 \end{array}\right]. \end{array}$$

The order of matrix multiplication results in different results, so it is necessary to specify the order of rotation, and the rotation order specified in Unity3D is *ZXY*. Therefore, the vector rotation in space is shown in the formula:

(9) $$\begin{array}{c} p^{\prime }=M_{RY}\cdot M_{Rx}\cdot M_{Rz}\cdot p. \end{array}$$

Among them, vector *p*^″^ is after the rotation.

In order to unify the coordinate expression, this paper uses homogeneous coordinates to express the translation transformation of the vector, as shown in formula (10) for the translation matrix *M*_*T*_:

(10) $$\begin{array}{c} M_{RT}=\left[\begin{array}{cccc} 1 & 0 & 0 & x_{t}\\ 0 & 1 & 0 & y_{t}\\ 0 & 0 & 1 & z_{t}\\ 0 & 0 & 0 & 1 \end{array}\right]. \end{array}$$

For the simpler scaling matrix of *k*-times space:

(11) $$\begin{array}{c} M_{S}=\left[\begin{array}{ccc} k & 0 & 0\\ 0 & k & 0\\ 0 & 0 & k \end{array}\right]. \end{array}$$

According to the above formula and following the principles of scaling, rotation, and translation, the transformation matrix *M*_*CW*_ from *O*_*C*_*X*_*C*_*Y*_*C*_*Z*_*C*_ to *O*_*W*_*X*_*W*_*Y*_*W*_*Z*_*W*_ can be obtained, and the transformation matrix *M*_*CW*_ is shown in the formula:

(12) $$\begin{array}{c} M_{CW}=M_{T}\cdot M_{RY}\cdot M_{RX}\cdot M_{RZ}\cdot M_{S}. \end{array}$$

When the operator operates on the screen, use the hand controller to control the displacement of the robot joint end. Assuming that the displacement of the joint end *O*_*C*_*X*_*C*_*Y*_*C*_*Z*_*C*_ in is *p*_*C*_ and the displacement in *O*_*W*_*X*_*W*_*Y*_*W*_*Z*_*W*_ is *p*_*W*_, *p*_*W*_ can be obtained from the formula:

(13) $$\begin{array}{c} p_{W}=M_{CW}\cdot p_{C}. \end{array}$$

In this paper, the movement of the joint end is based on *O*_*V*_*X*_*V*_*Y*_*V*_*Z*_*V*_, so it is necessary to use *O*_*V*_*X*_*V*_*Y*_*V*_*Z*_*V*_ to describe the displacement of the joint end under *O*_*W*_*X*_*W*_*Y*_*W*_*Z*_*W*_. Assuming that the displacement of the joint end in *O*_*V*_*X*_*V*_*Y*_*V*_*Z*_*V*_ is *p*_*V*_, *p*_*V*_ can be obtained from the formula:

(14) $$\begin{array}{c} p_{V}=M_{WV}\cdot p_{W}. \end{array}$$

Among them, *M*_*WV*_ is the conversion matrix from *O*_*W*_*X*_*W*_*Y*_*W*_*Z*_*W*_ to *O*_*V*_*X*_*V*_*Y*_*V*_*Z*_*V*_. Since the camera coordinate system and robot coordinate system are essentially local coordinate systems, *M*_*WV*_ is the inverse matrix of *M*_*CW*_. As mentioned earlier, the difference between the real robot coordinate system and the coordinate system in Unity3D is that the real robot coordinate system is the right-hand coordinate system. Therefore, it is necessary to convert the displacement in the left-hand coordinate system to the right-hand coordinate system. For the displacement in the virtual robot coordinate system, assuming that the joint end displacement in the real robot is expressed as *p*_*r*_, then *p*_*r*_ is obtained from the formula:

(15) $$\begin{array}{c} p_{r}=M_{lr}\cdot p_{v}. \end{array}$$

Among them, *M*_*lr*_ is the conversion matrix from the left-hand coordinate system to the right-hand coordinate system. The corresponding relation between the left-hand coordinate system and the coordinate axis of the right-hand coordinate system is obtained. *M*_*lr*_ is a fixed matrix in Unity3D, as shown in the formula:

(16) $$\begin{array}{c} \left[\begin{array}{cccc} -1 & 0 & 0 & 0\\ 0 & 0 & -1 & 0\\ 0 & 1 & 0 & 0\\ 0 & 0 & 0 & 1 \end{array}\right]. \end{array}$$

The above is a conversion process of the joint end vector from *O*_*C*_*X*_*C*_*Y*_*C*_*Z*_*C*_ to *O*_*r*_*X*_*r*_*Y*_*r*_*Z*_*r*_. The overall schematic diagram from the displacement of the joint end to the feedback received by the operator is shown in Figure 4.

RETRACTED

### 3.3. Wireless Sensor Networks (WSNs)

The communication software and hardware are responsible for communication and data transmission with other sensor points. With the help of WSNs, human beings can realize a more convenient ability to understand and know the objective world [16, 17]. WSNs network nodes have low-cost, self-distribution power supply and do not need the support of communication infrastructure. Therefore, they can also be self-organized into a network in some complex target environment areas to form effective monitoring of the target area. At present, WSNs have broad application prospects in medical care, environmental monitoring, traffic management, space exploration, industrial and agricultural production, military, and other fields [18–22]. With the further expansion of the depth and breadth of WSNs network application, it will have a great impact on people's production and life and promote another major change in society. The typical architecture of WSNs is shown in Figure 5.

The topology of WSNs is very dynamic [23]. However, there are also great differences between WSNs and traditional wireless ad hoc networks, which are mainly reflected in the following aspects: (1) limited node resources. Sensor nodes are generally powered by batteries. Due to the miniaturization of sensor nodes, the capacity of batteries is limited. In many sensor applications, nodes are deployed in areas with a poor environment, so it becomes very difficult or almost impossible to replace batteries manually. Therefore, the energy of nodes is very valuable because of their limitations. Because of the limited energy, how to improve the energy efficiency of nodes has become one of the important indicators of WSNs key technology design. In addition, due to the use of an embedded microprocessor, the processor capacity and memory size are limited, resulting in the limited computing and storage capacity of nodes, which also brings some challenges to the design of many key technologies of WSNs. (2) The network scale is large. Due to the limited function of a single sensor node, in order to better perceive the information of the monitoring area, it needs to deploy a large number of sensor nodes to make up for the limited function of a single node. In this way, it can not only improve the coverage of the network but also improve the accuracy of monitoring. However, the larger network scale brings some difficulties to the maintenance of the network. (3) The reliability of nodes is low. Because sensor nodes are often deployed in hostile or harsh environments, it leads to nodes working unattended. It makes it very difficult to maintain the node, which leads to the node being easy to damage or fail. Therefore, how to improve the self-reconfiguration ability of the network is a problem worthy of study. (4) It is data-centric. The main function of WSNs is to transmit the collected data to the sink node and then process it accordingly. When the user needs to query whether an event occurs in a certain area, the user does not care which node transmits the data but only whether the collected data indicates whether the event occurs or not. Because WSNs is a task-oriented network; users do not care about a node but only about the data related to the task. (5) High data redundancy. In many sensor network applications, nodes are randomly deployed in the monitoring area for data collection. This leads to the high similarity of the data collected by the nodes adjacent to the geographical location, that is, the data redundancy caused by spatial correlation. On the other hand, in a certain period of time, the value of the data collected by a single node changes little, which will also cause data redundancy, that is, data redundancy caused by time correlation. Therefore, how to remove redundant data without affecting the main functions of the network is an important challenge. (6) Application relevance: it is an obvious feature of WSNs different from other wireless networks. In the field of national defense and military affairs, the WSNs system pays more attention to the security and accuracy of data. In the field of public security, the WSNs system should minimize the false positive rate and false negative rate. In the field of target tracking, WSNs system pays more attention to the real-time monitoring of emergencies. In the field of health monitoring, more attention is paid to energy saving and protecting the privacy of monitored objects [24, 25]. It is precise because the characteristics of the WSNs are different from other wireless networks, which makes the design of some key technologies of WSNs face many challenges. The most important challenge is how to improve the energy efficiency of nodes when designing network protocols and data management algorithms [26, 27].

RETRACTED

## 4. Digital Twin Training Platform

In order to verify the rationality of the digital twin method described in this paper, this paper develops a digital twin platform for Brazilian jujitsu training. Based on the analysis of data integration requirements and the research on physical information fusion technology and data interaction technology, this paper designs a digital twin training platform and describes the development process of the platform in detail.

### 4.1. Design of Digital Twin Training Platform

A digital twin training platform is a complex training management and control platform composed of multiple systems. In order to facilitate real-time data acquisition, physical information fusion, data storage and transmission, visual monitoring, and online simulation of digital twin training, the platform is divided into 3 subsystems: OPCUA server, Demo3D visual simulation software, and general management system. In addition, as the basis for realizing digital twinning, the platform also needs to be extensible and extensible. By providing a data interface to cooperate with other application service systems, it can realize the functions of digital twinning, such as deduction, simulation, decision-making, and so on. The design idea of the digital twin training platform is shown in Figure 6.

1. Opcua server, the OPCUAserver of digital twin training, is the data transmission link between various systems. It is necessary to use the information modeling ability of OPCUAto realize physical information fusion and construct the OPCUA transmission service. OPCUA server is directly deployed in physical training, and its function is mainly divided into two parts. First, through the direct access or protocol conversion of manufacturing IOT equipment, it can realize the collection and data integration of full cycle, full element, and multidimensional data. It has the function of direct control over the production factors on the training site. The second is to import the OPCUA information model, bind the manufacturing IOT equipment to collect data, and complete the instantiation of the information model and the construction of address space so as to realize physical information fusion and information interaction and sharing with the other two subsystems based on the information model.
2. Demo3D visual simulation software Demo3D is a logistics simulation management and control system developed by the British Emulate3D company. It has the ability to import a geometric model, constructing a three-dimensional training structure and visual dynamic monitoring, and it can integrate the physical characteristics of entities into the geometric model to achieve a highly realistic training simulation effect. Therefore, it can build a virtual space of digital twin training based on Demo3D software and realize real mapping and online simulation through OPCUA client embedded in the software.
3. Overall management system: the overall management system can realize the overall planning and coordination of the other two subsystems. It saves the historical information of the whole platform through the data storage function and configuration management function and increases the scalability and flexibility of the platform so that managers can dynamically adjust the platform configuration according to the actual situation of the training site.

RETRACTED

Because the Demo3D software has the function of web page publishing, it can achieve a seamless connection with the overall management system through the URL link of the web page. So the whole digital twin training platform can be regarded as a system of B/S architecture. OPCUA server, general management system background, and Demo3D software can be regarded as the background program of the whole platform. The Demo3D visualization page and the overall management system interface can be used as the foreground interface of the platform.

The overall management system controls and coordinates the whole platform and other subsystems. This system mainly includes three functions: platform management, IOT equipment management, and OPCUAserver management. They are, respectively, used for the basic setting of the platform, configuration of manufacturing IOT equipment, and OPCUAserver in training.

The Demo3D software is used to construct the virtual training scene of the digital twin training platform. By utilizing the functions and advantages of Demo3D software in modeling and simulation, this paper integrates Demo3D software into the digital twin training platform to realize two functions of visual monitoring and training model management. Visual monitoring is to display all production activities on the training site in the form of three-dimensional visualization through the collected real-time data. At the same time, it pushes some production status information in real-time to realize the effect of virtual real mapping. Training model management is the process of constructing, configuring, and storing the virtual models corresponding to all production factors in virtual training. It plays the role of a physical object database in a digital twin training platform.

OPCUA server is the bottom data base of the whole platform. It is used to perceive the production status of the training site and realize physical information fusion and information transmission. OPCUA server mainly includes five functions: IOT equipment connection, physical information fusion service, address space service, information transmission service, and data interface service. IOT equipment connection is the process of connecting the manufacturing IOT hardware equipment deployed in physical training to the digital twin platform. It mainly includes the connection of equipment and the management of IP address, interface, and transmission protocol, which cooperate with the IOT equipment management function in the overall management system. It finally realizes the effective collection of multisource and multiprotocol data. The physical information fusion service is the realization of the physical information fusion method described above. Through the management of real-time data acquisition and control methods of production factors, as well as the steps of deredundancy, unit level fusion, spatial scale fusion, and training level fusion, it finally achieves the purpose of regulating heterogeneous factors and describing the whole training production state. Address space service is the representation of physical information fusion results in OPCUA server. Based on the information model imported from the overall management system, it instantiates the information model according to the physical information fusion process and constructs the address space model. Information transmission service is based on the construction of the address space model. It realizes data transmission based on TCP/IP protocol and provides subscription/connection function and method call function for OPCUA client. The data interface service provides the information exchange channel between the digital twin training platform and other application systems based on OPCUA.

RETRACTED

In order to meet the operational needs of training managers and maintain the convenience of platform development and deployment, this paper selects B/S architecture to develop this platform. For the OPCUA server, because it needs to connect with many hardware devices, and many devices do not directly support the OPCUA protocol, this paper needs to be written in a unified language to maintain a close relationship between the two. In addition, although OPCUA service software such as kepserver has appeared, due to the need to realize the physical information fusion process, the open source library of OPCUA must be used for server development.  Table 3 lists the OPCUAopen source libraries that are widely used at present. By comprehensively comparing the development data of various open source libraries in Table 3 and some existing hardware device development package languages, this paper selects open62541 based on C + + language as the development library of OPCUA server. Microsoft Visual Studio 2017 is the main development environment.

### 4.2. Deployment of Digital Twin Environment

RFID equipment consists of a reader, antenna, and passive tag. The reader/writer converts the current signal into an RF signal and radiates outward by connecting the antenna. When contacting the tag, the RF signal will be fed back to the tag itself. The antenna converts RF information into a current signal, and the reader and writer analyze and forward the signal.

RETRACTED

Considering practicability and economy, xc-rf807 fixed UHF RFID reader and xctf8421-c03 ceramic antimetal tag are selected for training. At the same time, it is in areas where RFID sampling frequency is not high, such as warehouse shelves. In this paper, xc-tx002 48 channel hub is used to reduce the number of readers and writers so as to reduce the cost. Different RFID antennas are required for different deployment environments. The training gate, entrance and exit, warehouse gate, and other areas need a huge antenna radiation range. Therefore, in this paper, we use the high power far field Valley XC-AF26 line polarization antenna. For the smaller areas, such as workstations and buffer areas, we use the XC-AF12-A remote circular antenna. For the smaller shelf space and the need to control the coverage area accurately, the KL12080 ultrahigh frequency ceramic antenna with smaller volume and smaller coverage is used. The physical drawing of RFID equipment is shown in Figure 7.

The virtual model includes three parts: geometric model, physical model, and logical model. It needs to import the three into Demo3D software, package them uniformly, and build a virtual model library. (1) The geometric model Demo3D software does not support direct modeling. It needs to use SolidWorks, ProE, and other three-dimensional modeling software to make real modeling of various production elements and training structures in training and save them into Demo3D software in the middle format. (2) The physical model is based on the geometric model of the imported production factors. By defining the function of the model attribute of the Demo3D software, the basic attributes of each production factor model and the dynamic variables of the control model change and mobile are defined. It realizes the physical model construction corresponding to the geometric model. (3) The logic model is based on the script writing function of Demo3D software, which uses the JScript language to write the logic script of the model. It realizes the connection with physical training and application services through OPCUAand database, realizes the evolution and simulation function of the logical model, and constructs the virtual model library.

### 4.3. System

For the digital twin environment, the real-time performance of data transmission and interaction is an important index to measure the performance of data interaction. There are still disputes about the maximum data transmission time delay acceptable for digital twin training. It is generally believed that the time delay from data collection to transmission to the data application module should be less than 20m [26, 28]. In order to verify the effectiveness of the information modeling method in this paper, it needs to model the information for the specific data acquisition node of physical training and build the corresponding OPCUA server and client. Because the data interaction between the OPCUA server and client has two transmission mechanisms: direct transmission and subscription, this paper uses different ways to test the delay time.

RETRACTED

The test uses Xeon E5 processor, 32g memory, and the service station of Windows Server 2016 system as the server of the data acquisition system. This paper uses a desktop computer with i7 processor, 12g memory, and Windows 10 system as the test client and uses a Gigabit switch to connect to the same LAN. During the test, this paper first constructs the OPCUA test server according to the OPCUA information modeling method. The test client is developed based on the OpcUaHelper Library Based on the C# language. Besides the normal functions of receiving, subscribing, sending, and so on, it also adds a simple time recording ability to the client. In addition, this paper establishes an OPCUA server without merging and adaptive compression of node data as the control group. It tests the effect of this scheme on improving the real-time performance of data acquisition.

In the virtual operation environment, the smooth running of the scene can not only reduce the dizziness of the operators but also make the operation look smoother so as to avoid the Caton problem caused by the tearing of the picture and effectively enhance the sense of presence. The FPS data in the experimental results are shown in Figure 8. It can be seen from the figure that although FPS will still fluctuate, the FPS using this method is the traditional method, which can achieve a more smooth training effect.

Under the direct transmission mechanism, the delay time of real-time data acquisition can be defined as the time from the client sending the request to receiving the data returned by the server and completing the analysis. The main factors affecting the data return time in the direct transmission mechanism are the data processing time and the data transmission time in Ethernet. Since the direct transmission mechanism is generally used to obtain the attribute data of production factors, this paper selects the attribute data node of material for the return time test. In the actual test, the test client sends a request to the server every 2 seconds and records the return time of 30 times in 1 minute. The results are shown in Figure 9.

The test results show that compression and merging can effectively reduce the return time of requests and reduce the time delay. Within one minute of the test, the average return time after treatment is 8.5 ms, and the maximum return time is 14.3 ms, both of which are less than the limit delay time of 20 ms.

RETRACTED

As shown in Figure 10, the test results are similar to those under the direct transmission mechanism. In the test process of 6 seconds, the average delay time is 5.2 ms, and the maximum delay time is 6.5 ms, both of which are less than the limit delay time of 20 ms. And compared with the control group, it achieved quite good results.

## 5. Conclusion

The cultural value of Brazilian jujitsu is reflected in three aspects. (1) The “melting pot” culture is embodied in Brazilian jujitsu. Brazilian jujitsu does not stick to one style and is good at learning from other technologies. While integrating the fighting technology of various countries, it also adds the cultural connotation of various countries to its own jujitsu system. It is not only a sport but also a representative of cultural integration. (2) The etiquette culture of Brazilian jujitsu. Although Brazilian jujitsu has not developed for a long time, it has always inherited the rigorous etiquette culture of Japanese traditional judo. It is very similar to Japanese judo in many places. (3) Brazilian jujitsu highlights the fighting culture. Through the confrontation of Brazilian jujitsu, people feel the Brazilian people's love for fighting. In this paper, the training system is studied, and the experimental results are also satisfactory. However, the article also has deficiencies. For example, in luansheng system, this paper selects too few joint points for human body simulation and can not simulate specific details. Therefore, in future research, it will also focus on more detailed twin simulations.

## Figures and Tables

**Figure 1:** Data twin reconfigurable system framework.

**Figure 2:** Schematic diagram of degrees of freedom of twin joint.

**Figure 3:** Schematic diagram of the hierarchical relationship of joints.

**Figure 4:** Data processing flow during operation.

**Figure 5:** Typical architecture of wireless sensor network.

**Figure 6:** Detailed functions of digital twin training platform.

**Figure 7:** Physical drawing of RFID equipment.

**Figure 8:** Comparison diagram of twin system FPS.

**Figure 9:** Experimental results of direct transmission mechanism.

**Figure 10:** Experimental results of platform delay.

**Table 1:** Corresponding joint angles.

Joint	*L*	*R*
1	0	0
2	−130	−130
3	30	30
4	0	0
5	40	40
6	0	0
7	135	135

**Table 2:** Range of joint motion.

Joint	Action type	Action level
1	Arm-rotational movement	−168.50 to +168.5°
2	Arm-bending exercise	−143.5° to +143.50
3	Flange rotation movement	−168.5° to +168.50
4	Flange rotation movement	123.5° to +80°
5	Leg_rotation movement	−290° to +290°
6	Leg_bending exercise	−88° to +138°
7	Foot-rotational movement	−229° to +229°

RETRACTED

**Table 3:** Common OPC UA open source libraries.

name	Programming language	Development platform	Type	Development information
Eclipse milo	Java	Windows, Linux	Client + server	Much
Node-opc-ua	JavaScript	Windows, Linux	Client + server	Many
open62541	C99	Windows, Linux	Client + server	Much
OpcUaHelper	C#	Windows	Client	Few
Opc Ua.NET	C#	Windows	Client + server	Few
FreeOpcUa	Python, C++	Windows, Linux	Client + server	Many

## Data Availability

The data that support the findings of this study are available from the corresponding author upon reasonable request.

## References

[1] Lee J. (2020). Integration of digital twin and deep learning in cyber-physical systems: towards. *Smart Manufacturing*.

[2] Li C., Mahadevan S., You L. (2017). Dynamic bayesian network for aircraft wing health monitoring digital twin. *AIAA Journal*.

[3] Hammoudeh M., Al-Fayez F., Lloyd H. (2017). A wireless sensor network border monitoring system: deployment issues and routing protocols. *IEEE Sensors Journal*.

[4] Zhao C., Wu C., Wang X. (2017). Maximizing lifetime of a wireless sensor network via joint optimizing sink placement and sensor-to-sink routing. *Applied Mathematical Modelling*.

[5] Lamonaca F., Carni D. L., Riccio M., Grimaldi D., Andria G. (2017). Preserving synchronization accuracy from the plug-in of NonSynchronized nodes in a wireless sensor network. *IEEE Transactions on Instrumentation and Measurement*.

[6] Edler J. R., Eberman L. E., Walker S. (2017). Clinical education in athletic training. *Athletic Training Education Journal*.

[7] Sniffen K. (2019). Embedding interprofessional activities with physical therapy and athletic training students in shared professional course. *International Journal of Health Sciences Education*.

[8] Bruce S., Crawford E., Wilkerson G., Dale R. B., Harris M., Rausch D. (2019). Prediction modeling for Board of Certification exam success for a professional master’s athletic training program. *Journal of Sports Medicine and Allied Health Sciences: Official Journal of the Ohio Athletic Trainers’ Association*.

[9] Yuri H. O. S. O. K. A. W. A. (2017). Exercise performance and safety in the heat. *Japanese Journal of Autogenic Therapy*.

[10] Roberts (2019). John. Mentorship and evidence based practice with athletic trainer preceptors: an overview. *Online Journal of Interprofessional Health Promotion*.

[11] Sridharan R., Domnic S. (2021). Placement for intercommunicating virtual machines in autoscaling cloud infrastructure. *Journal of Organizational and End User Computing*.

RETRACTED

[12] Sathiyamoorthi V., Keerthika P., Suresh P., Zhang Z., Rao A. P., Logeswaran K. (2021). Adaptive fault tolerant resource allocation scheme for cloud computing environments. *Journal of Organizational and End User Computing*.

[13] Baskaran N., Eswari R. (2021). Efficient VM selection strategies in cloud datacenter using fuzzy soft set. *Journal of Organizational and End User Computing*.

[14] Mansell J., Moffit D. M., Russ A. C., Thorpe J. N. (2017). Sexual harassment training and reporting in athletic training students. *Athletic Training Education Journal*.

[15] Sniffen K., Briggs E., Hinyard L., Breitbach A. (2019). Interprofessional role clarity, case-based learning, and perceptions of group effectiveness among athletic training and physical therapy students in a shared professional course. *The Internet Journal of Allied Health Sciences and Practice*.

[16] Lininger M. R., Riemann B. L. (2018). Statistical primer for athletic trainers: understanding the role of statistical power in comparative athletic training research. *Journal of Athletic Training*.

[17] Schilling J. (2017). Instructional strategy: didactic media presentation to optimize student learning. *Athletic Training Education Journal*.

[18] Khalaf O. I., Abdulsahib G. M. (2021). Optimized dynamic storage of data (ODSD) in IoT based on blockchain for wireless sensor networks. *Peer-to-Peer Networking and Applications*.

[19] Khalaf O. I., Abdulsahib G. M., Sabbar B. M. (2020). Optimization of wireless sensor network coverage using the bee algorithm. *Journal of Information Science and Engineering*.

[20] Abdulsahib G. M., Khalaf O. I. (2021). Accurate and effective data collection with minimum energy path selection in wireless sensor networks using mobile sinks. *Journal of Information Technology Management*.

[21] Khalaf O. I., Romero C. A. T., Hassan S., Iqbal M. T. (2022). Mitigating hotspot issues in heterogeneous wireless sensor networks. *Journal of Sensors*.

[22] Adil M., Song H., Ali J. (2022). EnhancedAODV: a robust three phase priority-based traffic load balancing scheme for internet of things. *IEEE Internet of Things Journal*.

[23] Smith-Ryan A. E., Hirsch K. R., Saylor H. E., Gould L. M., Blue M. N. M. (2020). Nutritional considerations and strategies to facilitate injury recovery and rehabilitation. *Journal of Athletic Training*.

[24] Kay M. C., Register-Mihalik J. K., Gray A. D., Djoko A., Dompier T. P., Kerr Z. Y. (2017). The epidemiology of severe injuries sustained by national collegiate athletic association student-athletes, 2009-2010 through 2014-2015. *Journal of Athletic Training*.

RETRACTED

[25] Register-Mihalik J., Baugh C., Kroshus E., Kerr Z., Valovich McLeod T. C. (2017). A multifactorial approach to sport-related concussion prevention and education: application of the socioecological framework. *Journal of Athletic Training*.

[26] Arnold A., Thigpen C. A., Beattie P. F., Kissenberth M. J., Shanley E. (2017). Overuse physeal injuries in youth athletes. *Sport Health: A Multidisciplinary Approach*.

[27] Driska A. P. (2020). Quality sport coaching in action: the application of the national standards for sport coaches in youth sport. *Strategies*.

[28] Stevens C. J., Mauger A. R., Hassmèn P., Taylor L. (2017). Endurance performance is influenced by perceptions of pain and temperature: theory, applications and safety considerations. *Sports Medicine*.

